# Screening Female Patients With Autonomic Nervous System Imbalance Using the Toho Medical Index Before Tooth Extraction

**DOI:** 10.7759/cureus.76345

**Published:** 2024-12-24

**Authors:** Kaoru Yamashita, Shusei Yoshimine, Akari Uto, Minako Uchino, Toshiro Kibe, Mitsutaka Sugimura

**Affiliations:** 1 Department of Dental Anesthesiology, Graduate School of Medical and Dental Sciences, Kagoshima University, Kagoshima, JPN; 2 Department of Oral and Maxillofacial Surgery, Graduate School of Medical and Dental Sciences, Kagoshima University, Kagoshima, JPN

**Keywords:** anxiety, autonomic imbalance, dental treatment, heart rate variability, toho medical index

## Abstract

Objective: Imbalanced autonomic nervous system (ANS) activity raises concerns about the development of systemic complications during dental treatment. The purpose of this study was to determine whether a psychological test (Toho Medical Index (TMI)) prior to the impacted mandibular third molar extraction can identify patients with potentially imbalanced autonomic function.

Materials and methods: In this prospective study, 34 healthy adult patients with no history of systemic disease were assigned to either the autonomic imbalance group (type II, III, IV) or the control group (type I) based on the results of the TMI. We evaluated sympathetic nervous system activity (low/high frequency (LF/HF)), parasympathetic nervous activity, heart rate (HR), and systolic blood pressure (SBP) values before extraction of the impacted mandibular third molar.

Results: LF/HF and SBP in the autonomic imbalance group were significantly higher preoperatively than those in the control group. In addition, preoperative HF values were significantly lower in the autonomic imbalance group compared to those in controls (Mann-Whitney U test, p < 0.05); no significant group differences in HR were found (Mann-Whitney U test, p < 0.05).

Conclusion: ANS activity before extraction of the impacted mandibular third molar was assessed subjectively using the TMI and objectively using HR variability analysis. Our findings suggest that some patients do not have symptoms specific to dysautonomia but have an imbalance of autonomic function before extraction of the impacted mandibular third molar, and TMI can identify such patients.

## Introduction

Dental treatment is often stressful for patients. Some people are unable to undergo dental treatment owing to associated anxiety [1-3]. Anxiety and tension related to dental treatment can cause fluctuations in autonomic nervous system activity (ANS), leading to medical emergencies such as elevated blood pressure (BP) and vasovagal reflexes [4-6]. The ANS is composed of the sympathetic and parasympathetic nervous systems (SNS and PSNS, respectively), and physical functions such as BP, respiration, digestion, and muscle tone become unregulated when the activities of these nervous systems are out of balance. In such an imbalance of ANS activity, one branch of the ANS predominates over the others, but the SNS is often increased and the PSNS is decreased, which is associated with a variety of pathologies [7]. Dental treatment of patients with dysautonomia who are at risk for fluctuating ANS activity raises concerns about the development of systemic complications. Therefore, it is important for dentists to understand a patient’s ANS activity before treatment to prevent systemic complications due to such fluctuations, which may lead to improved quality of intraoperative systemic management. The Toho Medical Index (TMI) is a questionnaire that combines autonomic symptoms and psychiatric symptoms to subjectively assess preoperative dysautonomia [1]. Heart rate variability (HRV) analysis is used as an objective measure to assess ANS activity and studies have attempted to visualize variations in ANS activity during dental treatment and oral surgery [8-15]. In HRV analysis, R-R interval frequency is analyzed and classified into low frequency (LF) and high frequency (HF); LF is derived from SNS and PSNS activity, while HF is derived from PSNS activity. As a result, the LF/HF ratio can be used as a measure of SNS activity and HF as a measure of PSNS activity [16]. To our knowledge, there have been no studies using both subjective and objective methods in the assessment of ANS activity before extraction of the impacted mandibular third molar.

We hypothesized that preoperative TMI would be useful in determining the state of a patient’s ANS activity. Among dental procedures, the extraction of an impacted mandibular third molar is one of the most stressful procedures for the patient [17-19]. Therefore, the aim of this study was to investigate whether administering the TMI prior to mandibular third molar extraction can screen patients with potential autonomic function imbalance.

The aim of this study was to determine whether ANS activity prior to extraction of the impacted mandibular third molar differs between patients with and without dysautonomia classified by the TMI. If preoperative TMI can screen patients with unbalanced autonomic function, dentists may be better prepared for unexpected medical emergencies.

## Materials and methods

Study design and ethical considerations

This study was a prospective observational study performed at Kagoshima University Hospital, Japan. This prospective study was conducted in accordance with the Declaration of Helsinki of the World Medical Association and was approved by the Kagoshima University Hospital Clinical Research Ethics Review Committee (approval number: 210062). Written informed consent was obtained from all participants.

Study criteria 

About 40 female patients aged 20 to 40 years with no history of systemic disease who were scheduled to undergo extraction of impacted mandibular third molars at our hospital between September 2021 and March 2022 were included in the study. Patients with diabetes, smoking, cardiovascular disease, impaired ANS, or a history of prescription medication use during the study period were excluded.

Procedure

Patients were instructed not to exercise or eat within 6 hours prior to HRV measurement, and the study started at 02:00 pm to minimize the influence of circadian rhythm [20-23]. Type I (normal) subjects were set as the control group, whereas the total of subjects with type II (autonomic imbalance), type III (psychosis), and type IV (psychogenic autonomic imbalance) were set as the autonomic imbalance groups, based on the TMI questionnaire. Patient examinations of HRV began with each patient seated in the supine position (room temperature, 24°C) on a dental chair, which was located in a noise-free private room. Patients completed the TMI questionnaire prior to treatment, and all patients were allowed to rest for 20 minutes before dental treatment began; preoperative HRV, heart rate (HR), and systolic blood pressure (SBP) were recorded, and the results were compared in two groups. Local anesthetics (2% lidocaine with 1:80,000 epinephrine) were infiltrated [24,25], and in all patients, the same oral surgeon performed impacted mandibular third molar extraction.

Assessment

Heart Rate Variability

The R-R interval was analyzed on electrocardiography using MemCalc-Makin2 (GMS, Tokyo, Japan), and HRV was calculated. The main frequency band of HRV consists of LF (0.04-0.15 Hz) and HF (>0.15 Hz) components; LF/HF and HF were, respectively, used as indicators of SNS and PSNS activity [9]. SBP was measured and analyzed non-invasively every 2 min. Resting ANS and circulatory data were sampled in the first 5 minutes after 15 minutes of rest following the start of rest [4,20,23].

Toho Medical Index

The TMI questionnaire included 43 questions regarding physical ANS symptoms and 51 questions regarding mental symptoms. The TMI questionnaire includes many psychosomatic symptoms and reflects psychosomatic autonomic imbalance. Type I (normal) included respondents who responded “yes” to ≤10 ANS symptoms and psychiatric symptoms; this is considered “normal” and indicates a stable state of the mind and body. Type II (autonomic imbalance type) included those who responded “yes” to ≥11 autonomic symptoms and ≤10 psychological symptoms; this is referred to as the autonomic imbalance type because it mainly involves autonomic symptoms. Type III (psychotic type) included those who responded “yes” to ≥11 psychotic symptoms and ≤10 ANS symptoms; psychotic symptoms are considered the main symptoms, and this type is called the psychotic type. Furthermore, type IV (psychopathic autonomic imbalance type) included those who responded with “yes” to ≥11 autonomic symptoms and psychological symptoms each.

Sample size calculation

The required sample size of 34 cases was estimated based on a power analysis (α = 0.05, β = 0.2, d = 1 SD) using G*power (University of Dusseldorf, Dusseldorf, Germany) and set at 40 to account for dropouts.

Statistical analysis

Data from the two groups were analyzed using GraphPad Prism 6 software (GraphPad Software, San Diego, CA). Comparisons between groups were made using the Mann-Whitney U test, with p < 0.05 being considered statistically significant.

## Results

Among the 40 eligible patients, six were excluded because they refused to consent to data collection. Thus, the data of 34 patients were analyzed. The autonomic imbalance group consisted of four type II (dysautonomic type) patients, six type III (psychotic type) patients, and seven type IV (psychogenic dysautonomic type) patients. The protocol is shown in Figure 1.

**Figure 1:** Description of the study protocol TMI: Toho Medical Index; HF: high frequency; LF: low frequency; HR: heart rate; SBP: systolic blood pressure

The control and autonomic imbalance groups each had 17 participants. There were no significant group differences in mean age, height, or weight of study participants (Table 1).

**Table 1:** Comparison of age, height, and weight between the control and autonomic imbalance groups Values are presented as mean ± standard deviation.

Data item	Control (n = 17)	Autonomic imbalance (n = 17)	Total (n = 34)	p-value
Age (years)	27.64 ± 8.1	29.94 ± 5.87	28.79 ± 7.06	0.19
Height (cm)	157.94 ± 5.43	157.09 ± 5.72	157.51 ± 5.51	0.68
Weight (kg)	47.82 ± 6.54	50.94 ± 8.22	49.38 ± 7.48	0.54

The participants’ extraction difficulty was classified as class II/position B based on Pell and Gregory’s classification [26]. Pre-autonomic nervous activities are shown in Figure 2.

**Figure 2:** Preoperative autonomic nervous system status (A) Low-frequency/high-frequency ratio (LF/HF); (B) high frequency (HF); (C) heart rate (HR); and (D) systolic blood pressure (SBP) values assessed during the rest period (analysis 1) are presented as mean ± standard error.

The LF/HF and SBP before surgery (analysis 1) were significantly higher in the autonomic imbalance group than in the control group (Figures 2A, 2D). HF values were significantly lower in the autonomic imbalance group than in the control group (Figure 2B). HR did not differ significantly between groups (Figure 2C). None of the patients experienced any medical emergencies during or after the surgery.

## Discussion

In this study, the TMI was used to detect patients with latent dysautonomic conditions that could not be detected during a routine medical interview. Patients classified as having dysautonomia suggested an imbalance in preoperative ANS activity, even in patients who were unaware of their dysautonomic symptoms. BP was elevated in the autonomic imbalance group compared to controls due to increased SNS activity and decreased PSNS activity; increased SNS activity may be associated with anxiety and nervousness about dental treatment [8,9,12-14]. In addition, ANS changes are briefly elicited by emotional changes, and except for the vasovagal reflex, PSNS activity decreases in response to stressful stimuli [27,28]. Thus, in this study, the decrease in PSNS activity may reflect stress from impending dental treatment. In this study, the TMI was able to detect potential dysautonomia, which was further supported by the results of HRV analysis. This study was targeted only for female patients, as it has been reported that dental phobia has more women [29]. The TMI used in this study was based on the Cornell Medical Index (CMI) developed by Brodman, Erdmann, and Woff at Cornell University in the United States, which was adapted for Japanese use by the Department of Psychosomatic Medicine of Toho University. The CMI was designed to investigate both mental and physical subjective symptoms of patients in a relatively short period of time and is widely used as a screening aid to determine the extent to which mental problems are involved as an adjunct to the clinical interview. The original CMI consists of 144 questions on somatosomatic symptoms and 51 questions on psychosomatic symptoms, for a total of 195 questions. Of the somatosomatic complaints, 43 were selected as those most likely to be manifested as complaints based on autonomic dysfunction, and 51 questions related to psychosomatic complaints were included to make a total of 94 questions for the TMI. Since the TMI contains fewer questions than the CMI, it is thought that patients were able to answer the questions more easily. Although there have been studies assessing patients’ ANS function before dental treatment [2,19,30], we have not found any studies using both subjective and objective methods, as in our study. Therefore, we believe the novelty of this study lies in the finding of the usefulness of obtaining TMI prior to the extraction of the impacted mandibular third molar.

The present study had limitations. In this study, type II (dysautonomia), type III (psychosis), and type IV (psychogenic dysautonomia) were evaluated together as the dysautonomia group, because a four-group comparison would require a large sample, and two groups were set up with the required sample size. Therefore, future research to capture the characteristics of each type is desirable. Future research is also needed to determine whether patients with a latent autonomic imbalance, which cannot be detected by interview, are more likely to develop systemic complications.

## Conclusions

In conclusion, we were able to assess ANS activity before extraction of the impacted mandibular third molar subjectively using the TMI and objectively using HRV analysis. It is suggested that some patients have no symptoms of dysautonomia but have an imbalance of autonomic function before extraction of the impacted mandibular third molar. TMI may be useful for screening such patients.

## Appendices

Appendix A

Autonomic Nervous Symptoms Survey Table

 Q1 Do you always have tinnitus?

 Q2 Have you ever had a feeling of tightness in your chest or heart?

 Q3 Have you ever felt like there was pressure on your chest or heart area?

 Q4 Do you often have palpitations that bother you?

 Q5 Does your heart often beat very fast?

 Q6 Do you often have difficulty breathing?

 Q7 Do you get short of breath more easily than others?

 Q8 Do you sometimes feel short of breath even when you are sitting down?

 Q9 Do your hands and feet get cold even in the summer?

 Q10 Do the tips of your hands and feet sometimes turn purple?

 Q11 Do you always have poor appetite?

 Q12 Do you have nausea or vomiting?

 Q13 Do you have stomach problems that bother you a lot?

 Q14 Do you have indigestion?

 Q15 Do you always have stomach problems?

 Q16 Do you have stomach pain after eating or when you are hungry?

 Q17 Do you often have diarrhea?

 Q18 Do you often have constipation?

 Q19 Do you have stiff shoulders or neck?

 Q20 Do you have tired legs?

 Q21 Do you have tired arms?

 Q22 Is your skin very sensitive and easily irritated?

 Q23 Does your face get very flushed?

 Q24 Do you sweat a lot in the winter?

 Q25 Do you often get hives on your skin?

 Q26 Do you often get severe headaches?

 Q27 Do you always have severe or painful headaches that bother you?

 Q28 Do you suddenly feel hot or cold?

 Q29 Do you often feel very dizzy?

 Q30 Do you ever feel faint or like you are going to collapse?

 Q31 Have you ever fainted more than twice?

 Q32 Do you have numbness or pain in any part of your body?

 Q33 Do you have tremors in your limbs?

 Q34 Do you sometimes sweat?

 Q35 Do you often feel tired and lazy?

 Q36 Do you feel very tired, especially in the summer?

 Q37 Do you feel tired when you work?

 Q38 Do you feel tired when you wake up in the morning?

 Q39 Do you feel tired after a short period of work?

 Q40 Do you ever feel so tired that you cannot eat?

 Q41 Does your physical condition change with changes in climate?

 Q42 Have you ever been told by a doctor that you have a peculiar constitution?

 Q43 Do you get motion sickness?

Mental Symptoms Survey Table

 Q1 Do you sweat or shake when you take an exam or are asked a question?

 Q2 Do you get very nervous and shake when a supervisor approaches you?

 Q3 Do you feel that you can't do your work at all when your supervisor is watching you?

 Q4 Do you often get confused when you have to do things in a hurry?

 Q5 Do you make mistakes easily when you are in a hurry?

 Q6 Do you always misunderstand instructions or orders?

 Q7 Do you feel anxious about strangers or places?

 Q8 Do you hesitate when you don't know someone?

 Q9 Do you always have trouble making up your mind?

 Q10 Do you always need someone to talk to?

 Q11 Do people think you are uncaring?

 Q12 Do you have difficulty eating in other restaurants?

 Q13 Do you feel alone and sad when you go to meetings?

 Q14 Do you feel unhappy and depressed all the time?

 Q15 Do you cry a lot?

 Q16 Do you always feel unhappy and depressed?

 Q17 Do you feel there is no hope in your life?

 Q18 Do you sometimes wish you were dead?

 Q19 Do you always worry?

 Q20 Do you have family members who worry about you?

 Q21 Do you worry about every little thing?

 Q22 Do people think that you are nervous?

 Q23 Do you have family members who are nervous?

 Q24 Have you ever suffered from severe neurosis?

 Q25 Do you have a family member with a severe neurosis?

 Q26 Have you ever been admitted to a mental hospital?

 Q27 Has anyone in your family ever been admitted to a mental institution?

 Q28 Do you have a severe shyor or nervousness?

 Q29 Do you have a family member with severe shyor nervousness?

 Q30 Are you easily upset?

 Q31 Do you get upset easily when people criticize you?

 Q32 Do people think you are difficult to deal with?

 Q33 Do people always misunderstand you?

 Q34 Do you feel uncomfortable around your friends?

 Q35 Do you feel like you can't stand still when you want to work?

 Q36 Do you get angry or irritated easily?

 Q37 Do you get upset easily when you are not always nervous?

 Q38 Do you get angry at the slightest thing that irritates you?

 Q39 Do you get angry when someone tells you what to do?

 Q40 Do you get angry when others annoy you?

 Q41 Do you get angry easily when you don't get your way?

 Q42 Do you get very angry?

 Q43 Do you often shake?

 Q44 Do you feel nervous and irritable all the time?

 Q45 Does a sudden noise make you jump or shake?

 Q46 Do you shrug when someone yells at you?

 Q47 Do you often hear sudden noises at night?

 Q48 Do you often wake up with frightening dreams?

 Q49 Do you often have frightening thoughts?

 Q50 Do you often break out in a cold sweat?
